# Modeling the Effect of Binding Kinetics in Spatial Drug Distribution in the Brain

**DOI:** 10.1155/2021/5533886

**Published:** 2021-07-05

**Authors:** Nelson Kashaju, Mark Kimathi, Verdiana G. Masanja

**Affiliations:** ^1^Department of Applied Mathematics and Computational Sciences, The Nelson Mandela African Institution of Science and Technology, P.O. Box 447, Arusha, Tanzania; ^2^Mathematics and Statistics Department, Machakos University, P.O. Box 136-90100, Machakos, Kenya

## Abstract

A 3-dimensional mathematical model is developed to determine the effect of drug binding kinetics on the spatial distribution of a drug within the brain. The key components, namely, transport across the blood-brain barrier (BBB), drug distribution in the brain extracellular fluid (ECF), and drug binding kinetics are coupled with the bidirectional bulk flow of the brain ECF to enhance the visualization of drug concentration in the brain. The model is developed based on the cubical volume of a brain unit, which is a union of three subdomains: the brain ECF, the BBB, and the blood plasma. The model is a set of partial differential equations and the associated initial and boundary conditions through which the drug distribution process in the mentioned subdomains is described. Effects of drug binding kinetics are investigated by varying the binding parameter values for both nonspecific and specific binding sites. All variations of binding parameter values are discussed, and the results show the improved visualization of the effect of binding kinetics in the drug distribution within the brain. For more realistic visualization, we suggest incorporating more brain components that make up the large volume of the brain tissue.

## 1. Introduction

The drug distribution is the process by which the drug molecules are delivered from the bloodstream to various body compartments, especially where the drug effect is needed [1]. The drug distribution in the human body is significant in a sense that it results into exposing the targeted sites to the drug being administered. However, drugs can only induce their therapeutic effects if they properly associate with the molecular targets within the body [2].

When the drug is administered to target the central nervous system, its distribution is usually varied due to various factors such as blood perfusion, permeability of the blood-brain barrier (BBB), diffusion, bulk flow of the brain extracellular fluid (ECF), metabolism, and drug binding [3, 4]. The delivery of drug substances into the brain is strongly controlled by the semipermeable brain border that is the BBB [5–7]. However, the ability of the drug to pass across the BBB largely depends on both biological features such as transporters and enzymes, as well as the drug compound physicochemical properties like molecular weight, lipophilicity, and hydrogen bonding capacity [8, 9].

The transport of drug molecules across the BBB may occur in two possible ways, which are either passive or active transport [10]. The study by Nhan et al. [11] describes passive transport across the BBB, in which this transport aspect exhibits bidirectional movement of drug compounds. Unlike the passive transport, active transport across the BBB exhibits the unidirectional movement of molecules from the blood to the brain. In active transport, the total flux across the BBB is similar to that of passive transport across the BBB and thus results into disregarding the unidirectional movement of molecules in the active transport across the BBB [12]. In addition, the total flux of the drug during active transport largely depends on the drug affinity, into and out of the brain [13]. However, the active transport is generally assumed to function as stated by Michaelis-Menten kinetics [14–17].

Drug molecules are normally exposed to both bulk flow of the brain ECF and drug diffusion into the brain ECF as they pass across the BBB [18, 19]. In the brain ECF, drug diffusion is constrained by the obstruction imposed by the substances and/or cells found within the brain ECF which result into a phenomenon known as tortuosity [20, 21]. Tortuosity is the diffusion property whereby diffusion is hindered by factors such as spaces occupied by brain cells as well as extracellular matrix. Furthermore, this property differs for different drugs due to their differences in size, drug deformability, and specific interactions of the drug with the extracellular matrix [22]. Since the brain ECF has a complex structure, it turns out that the diffusion of drug molecules via the brain ECF is lessened due to various factors like the hindrance imposed by the brain cells (tortuosity) and volume fraction of the brain ECF. However, in 2019, Vendel suggested that in order to account for the complex intertwined structure of the brain, the tortuosity and the brain ECF volume fraction should be taken into account in developed models [12]. Drug molecules need to be supplied to the specific targets in enough amounts and continuance to sufficiently interact together with the binding targets and elicit the desired effect [23, 24]. As a result, numerical understanding is greatly needed on binding positions and binding kinetics in the brain for suitable prediction of a drug effect [12]. Besides, the human brain is solely unavailable for experiments, and the instant measuring of the distribution of the drug within the brain's space is highly limited [12]. As a result, an extreme restriction is imposed on measuring the concentration-time profile of a drug within the brain. In this particular case, mathematical modeling becomes an essential tool for adequately forecasting the drug distribution within the brain and more significantly to depict and gain insights about the impact of processes that influence the distribution of the drug, especially those that occur within the brain [2, 12].

Currently, there are only few mathematical models that have been formulated and analyzed to study the drug distribution in the brain. These include a 2-dimension model by Vendel et al. [23] and 3-dimensional model by Vendel et al. [2] that incorporate blood-brain barrier (BBB), bulk flow of the brain extracellular fluid (ECF), drug diffusion through the brain extracellular fluid, and binding kinetics. However, the authors considered only the unidirectional bulk flow of the brain ECF. Therefore, this study intends to formulate and analyze a 3-dimensional mathematical model that incorporates the BBB, binding kinetics, and drug transport in the brain ECF with a bidirectional flow of the brain ECF to study what effect the drug binding kinetics imposes on the drug distribution in the brain. In addition, the study considers the bidirectional bulk flow of the brain ECF in order to capture the more realistic flow of blood within the brain unit which cannot be achieved with consideration of only one direction bulk flow of the brain ECF. Moreover, the study gives improved visualization of the drug distribution in the brain which leads into better understanding of the effect of the drug binding kinetics.

## 2. Materials and Methods

### 2.1. Model Assumptions and Model Formulation

The model formulation is based on the following assumptions:

- The drug concentration within the blood plasma is defined as a function of the rates of absorption and elimination from and into the blood. In this case, the drug is assumed to be orally administered into the body
- The drug is transferred into a 3-dimensional brain unit through a supplying arteriole, whereby it exits through a draining venule (see Figure 1(a))
- The drug enters a 3-dimensional brain unit at the *W*_in_ domain and leaves through the domain *W*_out_ (see Figure 1(b))
- The blood flow along capillaries of the brain is directed away from *W*_in_ (see Figure 1(c))
- Diffusion in the blood plasma is negligible; thus, drug molecules are exclusively transported by the brain capillaries via the brain capillary blood flow
- The brain capillaries are of all equal surface area and size. Besides, we assume that the volume of the incoming arteriole equals the volume of the three outgoing brain capillaries it connects to and that the volume of the outgoing venule equals the volume of the three incoming brain capillaries it connects to. Thus, the total volume of incoming blood vessels equals the total volume of the outgoing blood vessels at each vertex, while in all capillaries, the velocity of brain capillary blood flow is assumed to be the same
- The entire drug within the blood plasma is in an unbound state and therefore, it can pass across the BBB. Furthermore, the drug exchange between the blood plasma and the brain ECF is described by both passive and active transport across the BBB in both directions
- Drug within the brain ECF is transported through the brain ECF bulk flow and diffusion
- Tortuosity is taken into consideration to account for the obstruction imposed to diffusion by the brain cells
- The rectangular Cartesian coordinate system is used to indicate the direction of the bulk flow of the brain ECF. The brain ECF bulk flow is bidirectional. It is pointed in the *x*-direction and *z*-direction (see Figure 1(c)). Additionally, both the *x*-directed and *z*-directed bulk flows of the brain ECF are assumed to be the same
- The entire drug is distributed within the brain ECF where the extracellular binding sites are available
- The drug binding is reversible such that the total concentration of a drug in binding targets (nonspecific and specific targets) remains unchanged
- The nonspecific and specific targets are uniformly distributed over a 3-dimensional brain unit. Additionally, binding targets have constant positions
- The nonspecific and specific binding targets are external to the cells. Thus, the drug does not cross the cell membranes to attach to the desired targets

Consider the figure above for reference.

### 2.2. Description of 3-Dimensional Brain Unit

In the model developed in the current study, a 3-dimensional brain unit is the domain under consideration. It is defined as

(1) $$\begin{array}{c} W=\left\{\left(x,y,z\right)\in \text{I}R^{3}\;|\;0\leq x\leq x_{r}\wedge 0\leq y\leq y_{r}\wedge 0\leq z\leq z_{r}\right\}, \end{array}$$

whereby *x*_*r*_, *y*_*r*_, and *z*_*r*_ stand for the length of one unit of the brain capillary, given by *l*_cap_ + 2*r* with *l*_cap_ as the intercapillary distance, and *r* is the radius of brain capillary.

Since the BBB, brain ECF and the brain capillaries are found in the brain; then, they are the subsets of one unit of the brain [2]. That is, *W*_*pl*_ ⊂ *W*, *W*_BBB_ ⊂ *W*, and *W*_ECF_ ⊂ *W*. Therefore, the domain of a 3-dimensional brain unit can be defined as

(2) $$\begin{array}{c} W=W_{\text{pl}}\cup W_{\text{BBB}}\cup W_{\text{ECF}}. \end{array}$$

The distribution of drug in the developed model is described by two main subprocesses, namely, the distribution of drug into the blood plasma and drug distribution in the ECF brain. This is shown in the system of differential Equations (4), (6), (7), and (8) along with the associated initial conditions described in Equations (5), (9), and (10) as well as the boundary conditions described in Equations (12) to (16).

### 2.3. Flow of Drug Concentration in Blood Plasma

As stated in assumption (i), i.e., the drug is assumed to be orally administered. Thus, the unbound drug concentration in *W*_in_ is expressed through Equation (3).

(3) $$\begin{array}{c} \mu {\left(t\right)}_{W_{\text{in}}}=\frac{F.\text{Dose}.K_{a}}{V_{d}\left(K_{a}-K_{e}\right)}\left(e^{-K_{e}t}-e^{-K_{a}t}\right), \end{array}$$

whereby *F* is the drug bioavailability, *μ* is the drug concentration within the blood plasma, Dose is the orally delivered drug concentration, *V*_*d*_ is the distribution volume that relates the drug concentration in the blood plasma with the total drug amount in the body, and *K*_*a*_ and *K*_*e*_ are the drug absorption and elimination constants, respectively.

Moreover, according to assumptions (iv) and (v), the equations governing flow of drug concentration in blood plasma are given by the system of Equations (4) and (5).

(4) $$\begin{array}{c} \begin{array}{c} \frac{\partial \mu }{\partial t}=-v_{\text{blood}}\frac{\partial \mu }{\partial x},\mu \in W_{xi},\forall_{i}\;|\;i=1,\cdots ,4,\\ \frac{\partial \mu }{\partial t}=-v_{\text{blood}}\frac{\partial \mu }{\partial y},\mu \in W_{yi},\forall_{i}\;|\;i=1,\cdots ,4,\\ \frac{\partial \mu }{\partial t}=-v_{\text{blood}}\frac{\partial \mu }{\partial z},\mu \in W_{zi},\forall_{i}\;|\;i=1,\cdots ,4. \end{array} \end{array}$$

The associated initial condition is

(5) $$\begin{array}{c} \mu \left(x,y,z,t=0\right)=0, \end{array}$$

where *v*_blood_ is the blood flow rate in the brain capillaries. *W*_*xi*_, *W*_*yi*_ and *W*_*zi*_, and ∀_*i*_ | *i* = 1, ⋯, 4 represent the directions of brain capillaries in *x*, *y*, and *z* directions, respectively.

### 2.4. Drug Distribution within the Brain ECF

Based on assumptions (viii) to (xiv), the distribution of both bound and unbound drugs within *W*_ECF_ is described in Equations (6) to (8).

(6) $$\begin{array}{c} \frac{\partial \rho }{\partial t}=\frac{D}{\lambda^{2}}\nabla^{2}\rho -v_{\text{ECF}}\left(\frac{\partial \rho }{\partial x}+\frac{\partial \rho }{\partial z}\right)-k_{1\text{on}}\rho \left(B_{1}^{tot}-B_{1}\right)+k_{1off}B_{1}-k_{2\text{on}}\rho \left(B_{2}^{tot}-B_{2}\right)+K_{2\text{off}}B_{2}, \end{array}$$

(7) $$\begin{array}{c} \frac{\partial B_{1}}{\partial t}=k_{1\text{on}}\rho \left(B_{1}^{\text{tot}}-B_{1}\right)-k_{1\text{off}}B_{1}, \end{array}$$

(8) $$\begin{array}{c} \frac{\partial B_{2}}{\partial t}=k_{2on}\rho \left(B_{2}^{tot}-B_{2}\right)-K_{2off}B_{2}. \end{array}$$

The associated initial conditions are

(9) $$\begin{array}{c} \rho \left(x,y,z,t=0\right)=0, \end{array}$$

(10) $$\begin{array}{c} B_{i}\left(x,y,z,t=0\right)=0,\forall_{i}\;|\;i=1,2, \end{array}$$

whereby *D* is the diffusion coefficient in a free medium, *λ* is the tortuosity, *ρ* is the concentration of drug in the brain ECF, and *v*_ECF_ is the (*x*-directed and *z*-directed) brain ECF bulk flow [20]. Furthermore, *B*_2_ and *B*_1_ are the drug concentrations in both nonspecific binding and specific binding targets, respectively, and *B*_1_^tot^ and *B*_2_^tot^ are the total concentrations of specific binding and nonspecific binding sites within the brain ECF, respectively [23]. Also, *k*_1on_ and *k*_2on_ are the association rate constant for both specific binding and nonspecific binding, respectively, where *k*_1off_ and *k*_2off_ are the dissociation rate constant for both specific and nonspecific binding, respectively [23]

### 2.5. Boundary Conditions

The system of equations above specifically Equations (3), (4), (6), (7), and (8) along with their associated initial conditions forms a mathematical model for this study. All of these equations describe the process of drug distribution over different subdomains within a 3-dimensional brain unit domain.

To manage the solving of model equations, it is important to specify realistic boundary conditions for this model. Such boundaries are boundaries at the faces of the brain unit, the boundary between the brain capillaries domain (*W*_pl_), and the brain-ECF domain (*W*_ECF_), i.e., at *x* = *r* and *x* = *x*_*r*_ − *r* (see Figure 2).

The diffusion of a drug from the blood plasma into the brain ECF is described as a product of the difference in concentration of drug between *W*_*pl*_ and *W*_*E*_CF and the BBB permeability.

Furthermore, based on the study in [2], drug transport in and out of the brain is described by Equation (11)

(11) $$\begin{array}{c} \begin{array}{c} f\left(\mu ,\rho \right)=P\left(\mu -\rho \right)+\frac{T_{m-\text{in}}}{\text{S}{\text{A}}_{\text{BBB}}\left(K_{m-\text{in}}+\mu \right)}\mu -\frac{T_{m-\text{out}}}{\text{S}{\text{A}}_{\text{BBB}}\left(K_{m-\text{out}}+\rho \right)}\rho \\ \text{With};P=p_{\text{trans}}f_{\text{trans}}+p_{\text{para}}f_{\text{para}}\text{ where }p_{para}=\frac{D_{\text{para}}}{W_{PCS}} \end{array}, \end{array}$$

where *p*_trans_ is the permeability across the endothelial cells of brain capillary, *f*_trans_ is the fraction of the area of endothelial cells of brain capillary, *D*_para_ is the diffusivity of a drug across the paracellular space, *W*_PCS_ is the breadth of the paracellular space, *f*_para_ is the fraction of area of the paracellular space, the maximal rates of active influx and active efflux of drug are given by *T*_*m*−in_ and *T*_*m*−out_, respectively, *K*_*m*−in_ is the concentration of drug where half of *T*_*m*−in_ is attained, *K*_*m*−out_ is the concentration of drug where half of *T*_*m*−out_ is attained, and SA_BBB_ represents the surface area of the BBB [2].

As Figure 2 indicates, the loss or gain of unbound drug from/into the brain ECF due to the BBB is described by the boundary conditions given by Equation (12) [23]:

(12) $$\begin{array}{c} \begin{array}{c} D^{*}\frac{\partial \rho }{\partial t}=-f\left(\mu ,\rho \right)\text{for }\left(x,y,z\right)\in W_{\text{BBB}}\;at\;x=r,\\ D^{*}\frac{\partial \rho }{\partial t}=f\left(\mu ,\rho \right)\text{for }\left(x,y,z\right)\in W_{\text{BBB}}\;at\;x=x_{r}-r. \end{array} \end{array}$$

Moreover, in view of the brain capillaries domain, the drug transport across the BBB is described by Equation (13):

(13) $$\begin{array}{c} \begin{array}{c} D^{*}\frac{\partial \mu }{\partial t}=f\left(\mu ,\rho \right)\;\text{for }\left(x,y,z\right)\in W_{\text{BBB}}\;at\;x=r,\\ D^{*}\frac{\partial \mu }{\partial t}=-f\left(\mu ,\rho \right)\;\text{for }\left(x,y,z\right)\in W_{\text{BBB}}\;at\;x=x_{r}-r, \end{array} \end{array}$$

where *D*^∗^ = *D*/*λ*^2^, *D*^∗^, is the effective diffusion coefficient while *D* is the coefficient of diffusion in free medium.

Additionally, considering assumption (v), i.e., there is no diffusion in blood plasma. It follows that the system of Equation (14) is used for description of the concentrations at the sides of 3-dimensional brain unit:

(14) $$\begin{array}{c} \begin{array}{c} \frac{\partial \mu }{\partial x}=0\;\text{for }x=0\text{ and }x=x_{r},\\ \frac{\partial \mu }{\partial y}=0\;\text{for }y=0\text{ and }y=y_{r},\\ \frac{\partial \mu }{\partial z}=0\;\text{for }x=0\text{ and }z=z_{r}. \end{array} \end{array}$$

In the model developed in the current study, concentration at the faces of 3-dimensional brain unit is considered to be zero as shown in Equation (15):

(15) $$\begin{array}{c} \mu =0\;\text{for }W_{\text{out}}\cap \partial W. \end{array}$$

Furthermore, the conditions at boundaries (*W*_ECF_∩*∂W*) are given by equations below:

(16) $$\begin{array}{c} \begin{array}{c} \frac{\partial \rho }{\partial x}=0\\ \frac{\partial \rho }{\partial z}=0 \end{array} \end{array}$$

## 3. Description of Model Parameters

In the current study, properties of the rat brain were used to determine the parameter values. This choice is made on the basis that most data for this species are available. Nevertheless, the model is suitably valid for data from human and other species [2]. The brain intercapillary distance in the rat is averagely considered to be 50*μm*, whereby the brain capillary is approximately 2.5*μm* by radius ([25–27]). It follows that the radius of capillaries in the brain, *r*, was set to 2.5*μm*,and the dimensions of the 3-dimensional brain unit in the directions of *x*, *y*, and *z* to 55*μm*.

Additionally, Equations (4) and (5) are used to describe concentration of the drug in blood plasma, and the boundary conditions are described by Equations (13), (14), and (15). We also describe the concentration of drug within the brain ECF through Equations (6), (7), and (8) and the initial conditions (9) and (10) along with boundary conditions described in Equations (12) and (16). The parameter values together with their units are given in Table 1. The choice of values for model parameters is based on the findings of different experimental studies.

## 4. Model Results

The drug distribution in the 3-dimensional brain unit is studied by plotting the concentration of drug in the blood plasma, drug binding sites, and the brain extracellular fluid for various time instances. The main focus of the current study is to determine the effect that the binding kinetics of drug imposes on the distribution of drug in the brain tissue. To determine the effect of drug binding kinetics, the model Equations (4), (6), (7), and (8) are discretized together with the prescribed boundary conditions (12), (13), (14), and (16). The discretization is done by using the finite difference method (FDM), particularly the implicit schemes through which the simulation is carried out. For improved visualization of the effect of drug binding kinetics, the drug distribution incorporated with drug transport across the BBB, binding kinetics of drug, and bidirectional bulk flow of the brain ECF is considered. The parameter values in Table 1 are used for simulation.

The blood flow within brain capillaries aids the movement of drug molecules within a 3-dimensional brain unit. The drug molecules within blood plasma have to cross the BBB for them to enter the brain ECF. The drug molecules bind either to nonspecific or specific binding targets in the brain ECF. In addition, the effect of binding kinetics is determined by studying the trends of how the drug distributes in the brain ECF. The drug transport process within the brain unit is described by Figure 3(a). Moreover, the cubical lattice in Figure 3(b) represents the 3-dimensional brain unit within which the brain ECF is found. In the simulations of the current study on how the drug distributes within the brain ECF, the cubical lattice in Figure 3(b) is sliced at different positions into three slices plots so as the effect of binding kinetics and concentration within the brain ECF can be easily observed at different time levels.

### 4.1. Drug Distribution in Blood Plasma

The unbound drug in the plasma has to pass through the BBB into the brain ECF where its therapeutic effect is determined. We firstly need to determine how the drug concentration distributes along the brain capillaries across the BBB into the brain ECF. The distribution is observed at three different levels of time *t*_1_ = 2sec, *t*_2_ = 8sec, and *t*_3_ = 14sec. Drug molecules leave the blood plasma domain across the BBB into the brain ECF where the drug molecules bind to either specific or nonspecific binding sites. The amount of unbound drug from blood plasma into the brain ECF is slightly affected by the permeability of BBB, *P*, and blood flow rate, *v*_blood_. Figures 4–7 show how the drug molecules distribute in the blood plasma when different cases of variations in the blood flow rate, *v*_blood_, and permeability of BBB, *P*, are considered. The model parameter values for permeability (*P* = 0.1 × 10^−7^*ms*^−1^) and blood flow rate (*v*_blood_ = 1 × 10^−6^*ms*^−1^) are initially used in the simulations for Figure 4 to describe how the drug distributes along brain capillaries into the brain ECF.

The plots in Figure 4 show that the concentration of drug within blood plasma slightly distributes within brain capillaries in significantly smaller amounts at different time levels for the mentioned permeability and blood flow velocity values. However, in Figure 5, the concentration of unbound drug within blood plasma appears to become considerably large when the BBB permeability and blood rate values are simultaneously increased, i.e., (*P* = 0.5 × 10^−7^ms^−1^) and (*v*_blood_ = 1.5 × 10^−6^ms^−1^). This implies that when the values for both BBB permeability and blood flow rate are increased simultaneously, the molecules of unbound drug within the blood plasma are found to have huge amount as seen in Figure 5(a). However, as time passes, the drug distributes further, and the concentration within the blood plasma becomes much more lesser due to elimination to the brain ECF. Thus, the concentration of drug within blood plasma tends to decrease as shown in Figures 5(b) and 5(c). Moreover, in Figure 5, when the BBB permeability (*P*) and blood flow rate (*v*_blood_) are simultaneously increased, the concentration of unbound drug in blood plasma is as much as a square of the concentration of drug in blood plasma for smaller values of BBB permeability (*P*) and blood flow rate (*v*_blood_) in Figure 4.

Nevertheless, the plots in Figure 4 exhibit spatial variations in the location of the drug concentration peaks in distribution of drug within the blood plasma at three different time levels. The variation of drug concentration peak within the blood plasma is initially observed at *t*_1_ = 2sec as indicated in Figure 4(a). The concentration peak in Figure 4(a) covers a small area contrary to Figures 4(b) and 4(c). When the time increases to *t*_2_ = 8sec, the concentration peak also spreads a little wider as shown in Figure 4(b). Additionally, when the time increases further to *t*_3_ = 14sec, the concentration peak within the blood plasma spreads more over the region next to the BBB as indicated in Figure 4(c).

The observation is further done to determine how the variations in individual parameter values of the BBB permeability (P) and blood flow rate (*v*_blood_), respectively, affects the distribution of drug within the blood plasma. The variation is done in one parameter value while another parameter value is kept constant as shown in Figures 6 and 7. Initially, the value for BBB permeability (*P*) is set to *P* = 2 × 10^−6.9^ms^−1^ while the blood flow rate is held constant, *v*_blood_ = 1 × 10^−6^ms^−1^. Thereafter, the blood flow rate is varied to *v*_blood_ = 1.1 × 10^−5.95^ms^−1^ while the BBB permeability is held constant, *P* = 0.1 × 10^−7^ms^−1^.

When the BBB permeability increases while blood flow rate is held constant, the concentration of unbound drug becomes less in the blood plasma.  Figure 6 shows that drug concentration within the blood plasma is slightly distributed in small amounts. Nevertheless, in a case when the blood flow rate is increased while the BBB permeability is held constant, an increased drug concentration within the blood plasma is observed as shown in Figure 7. Moreover, spatial variations in drug concentration peak in Figures 6 and 7 are observed at different time levels. In Figures 6(a) and 6(b), the drug distribution within the blood plasma is approximately the same for the first two time levels, i.e., *t*_1_ = 2sec and *t*_2_ = 8sec; however, the distribution of drug tends to increase in the region next to the BBB as time increases due to the increased permeability as shown in Figure 6(c). Additionally, in Figure 7(a), the drug distribution within the blood plasma is observed to be less compared to that observed in Figure 7(b), but as time goes on, the drug distribution in the blood plasma tends to decrease to a minimal drug concentration due to elimination of drug from the blood plasma, Figure 7(c).

### 4.2. The Effect of Binding Kinetics in Drug Distribution within a 3-Dimensional Brain Unit

After crossing the BBB, the drug molecules diffuse into the brain intercellular spaces and distribute throughout the brain ECF via the bulk flow of the brain ECF. However, the distribution of free drug molecules in the brain ECF is somewhat affected by the binding kinetics of the drug at their binding targets. Therefore, it is important to determine how the binding kinetics of drug affects the drug distribution within the brain.

Both diffusion and bulk flow of a drug result into a substantial amount of drug concentration within the brain ECF. This maximizes the chances of drug molecules to associate with either specific or nonspecific binding targets. Moreover, the chance for drug binding kinetics to induce its effect on the drug distribution within the brain ECF becomes higher.

The impact of drug binding kinetics is determined through investigating the trends of distribution of a free drug within the brain ECF at three distinct time levels (*t*_1_ = 2sec, *t*_2_ = 8sec, and *t*_3_ = 14sec) when different values for drug association and dissociation rates (*k*_*i*on_ and *k*_*i*off_, respectively, for *i* = 1, 2) are considered in the simulated plots (see Figures 8–12).

First, we consider a case where the model is simulated by fixed parameter values of binding kinetics to see how the drug distributes within the brain ECF, as indicated in Figure 8. Thereafter, simulation for different cases of variations in the binding parameters (see Figures 9–12) is considered to see how the distribution of drug within the brain is affected.

Initially, values for binding kinetics are fixed with *k*_1on_ = 1 × 10^−1^(*μ*molL^−1^*s*)^−1^, *k*_2on_ = 1 × 10^−2^(*μmol*L^−1^*s*)^−1^, *k*_1off_ = 1 × 10^−2^*s*^−1^, and *k*_2off_ = 1 × 10^−1^*s*^−1^ for Figure 8. The drug molecules in the region of the brain ECF adjacent to the BBB distribute in huge amounts throughout the whole region next to the BBB for the first level of time (*t*_1_ = 2sec) (see Figure 8(a)). At the second time level (*t*_2_ = 8sec) as indicated in Figure 8(b), drug molecules distribute with a slight decrease in drug concentration within the brain ECF. Figure 8(b) shows that drug concentration within the brain ECF decreases over almost the whole region of the brain ECF except a very few areas where the concentration is a bit higher. However, when the time further increases in Figures 8(c) and 8(a), significant decrease in amount of the drug concentration within the brain ECF is noticed. Thus, the drug concentration in Figure 8(b) is less compared to Figure 8(a) but reasonably higher compared to the concentration when time increases further to *t*_3_ = 14sec as indicated in Figure 8(c).

In this case, the association rate in specific binding is the same as the dissociation rate in nonspecific binding sites. Nevertheless, the association rate in nonspecific binding is the same as the dissociation rate in specific binding. The association rate at specific binding sites is larger compared to that at nonspecific sites; hence, the drug molecules associate fast with the specific sites as compared to the nonspecific sites. Moreover, the dissociation rate at nonspecific binding sites is larger compared to the one at specific binding sites. This results into high dissociation of the drug at nonspecific binding sites. Therefore, the drug distributes in nonspecific binding sites with slightly large amount of concentration than in specific binding targets, (see Figures 13 and 14).

#### 4.2.1. Impact of Varying Dissociation Rates (*k*_1,2off_) while Maintaining Association Rates (*k*_1,2on_)

The effect of drug binding kinetics, (*k*_*i*on_ and *k*_*i*off_, for *i* = 1, 2), on the drug distribution within the brain with variations in dissociation rates is further assessed. In this particular case, the association rate of specific binding sites (*k*_1on_ = 1 × 10^−1^(*μmol*L^−1^*s*)^−1^) is larger than the association rate at nonspecific binding sites (*k*_2on_ = 1 × 10^−2^(*μ*molL^−1^*s*)^−1^). Also, the dissociation rate at nonspecific binding sites (*k*_2off_ = 3 × 10^−0.2^*s*^−1^) is larger than the dissociation rate at specific binding sites (*k*_1off_ = 5 × 10^−1^*s*^−1^).

Initially at (*t*_1_ = 2sec), the concentration of drug in the brain ECF region next to the BBB is found to be considerably large and spread widely over that region (see Figure 9(a)). Nevertheless, drug molecules within the brain ECF continue to spread with a slight decrease in concentration as time increases to (*t*_2_ = 8sec) (see Figure 9(b)). Moreover, the concentration of drug tends to diminish to a lesser amount as time increases further to (*t*_3_ = 14sec), as shown in Figure 9(c). Thus, in Figures 9(a) and 9(b), the concentration of drug within the brain ECF at the first two-time levels exhibits a gradual decrease over the whole region of the brain ECF. Additionally, as the time further increases in Figure 9(c), the drug concentration within the brain ECF becomes much more lesser due to absorption within the brain ECF. However, the drug concentration amount in the brain ECF for both Figures 8 and 9 is almost the same.

Contrary to when small values of dissociation rates are considered in Figure 8, the drug molecules in Figure 9 distribute more widely over the brain ECF region due to higher dissociation of drug molecules. Furthermore, the drug concentration in nonspecific binding sites (see Figure 15) is slightly more compared to the concentration in the specific binding targets (see Figure 16).

#### 4.2.2. Impact of Varying Association Rates (*k*_1,2on_) while Maintaining Dissociation Rates (*k*_1,2off_)

The effect of binding kinetics is also observed when the drug association rates are varied. With varied association rates, the drug molecules within the brain ECF do not spread widely even though the concentration within the brain ECF is considerably high compared to that in the binding sites, both specific and nonspecific. Moreover, drug concentration in the nonspecific binding sites is significantly large compared to that found in the specific binding sites.

The effect of change in association rates while maintaining the drug dissociation rates is assessed. The association rate in specific binding sites (*k*_1on_ = 1 × 10^−2^(*μ*molL^−1^*s*)^−1^) is greater than the one at nonspecific binding sites (*k*_2on_ = 1 × 10^−3^(*μ*molL^−1^*s*)^−1^). In addition, the dissociation rate at the specific binding sites (*k*_1off_ = 1 × 10^−2^*s*^−1^) is less than the one at nonspecific binding sites (*k*_1*off*_ = 1 × 10^−1^*s*^−1^). Simulation results show an increased concentration amount in nonspecific binding sites (see Figure 17) compared to the specific binding sites (see Figure 18). Nevertheless, the distribution of drug concentration in the brain ECF slightly change with time in considerably small amount.

In addition, spatial variations of the location of drug concentration peak are observed in Figure 10. Initially at *t*_1_ = 2sec, the drug concentration peak within the brain ECF is observed in a region near *W*_in_ as indicated in Figure 10(a). Moreover, the concentration peak in Figure 10(a) covers a small area unlike in Figures 10(b) and 10(c). When the time increases to *t*_2_ = 8sec, the concentration peak also spreads a little bit more as shown in Figure 10(b). Moreover, when the time is further increased to *t*_3_ = 14sec, the concentration peak within the brain ECF spreads more over the region of the brain ECF in the direction of *W*_out_ as indicated in Figure 10(c). Thus, the concentration peaks of drug within the brain ECF are found to cover different locations over the region when the association rates are altered. In addition, the drug molecules distribute within the brain ECF with an increasing pattern as time also increases.

#### 4.2.3. Impact of Varying both Association and Dissociation Rates, (*k*_1,2on_) and (*k*_1,2off_) Simultaneously

We then look on how simultaneous variations in both association and dissociation rates affect the distribution of drug within the brain ECF. In Figure 11, we first make the alteration in both association rate and dissociation rates for specific binding sites (*k*_1on_ = 0.5(*μ*molL^−1^*s*)^−1^ and *k*_1off_ = 2 × 10^−1^*s*^−1^, respectively) while the association and dissociation rates for nonspecific remain unchanged (*k*_2on_ = 1 × 10^−2^(*μ*molL^−1^*s*)^−1^ and *k*_2off_ = 1 × 10^−1^*s*^−1^, respectively). Thereafter, the association and dissociation rates for nonspecific binding sites are varied with values (*k*_2on_ = 2.5 × 10^−4^(*μ*molL^−1^*s*)^−1^ and *k*_2off_ = 1.5 × 10^−3^*s*^−1^, respectively) while maintaining those for specific binding sites i.e. (*k*_1on_ = 1(*μ*molL^−1^*s*)^−1^ and *k*_1off_ = 1 × 10^−2^*s*^−1^, respectively), for Figure 12. Simulation results for Figure 11 show that drug distributes widely within the region of the brain ECF for the first two-time levels (*t*_1_ = 2sec and *t*_2_ = 8sec) with significantly small concentration as indicated by Figures 11(a) and 11(b). However, there is a gradual change in the coverage of drug molecules in Figures 11(a) and 11(b) whereby the drug molecules decrease significantly in relation to an increase in time. Nonetheless, the results in Figure 11(c) show a higher decrease in amount of drug molecules within the brain ECF when the time increases further to *t*_3_ = 14sec.

Contrarily, the results in Figure 12 show that the drug distributes over the brain ECF region with spatial variations in the location of the concentration peaks. The spatial variations of the location of drug concentration peak in Figure 12 are initially observed at *t*_1_ = 2sec. The drug concentration peak within the brain ECF at *t*_1_ = 2sec is observed in a region near *W*_in_ as indicated in Figure 12(a). Moreover, the concentration peak in Figure 12(a) covers a small area unlike in Figures 12(b) and 12(c). When the time increases to *t*_2_ = 8sec, the concentration peak also spreads a little wider as shown in Figure 12(b). Additionally, when the time increases further to *t*_3_ = 14sec, the concentration peak within the brain ECF spreads more over the region of the brain ECF in the direction of *W*_out_ as indicated in Figure 12(c). Thus, the concentration peaks of drug within the brain ECF are found to cover different locations over the region when the association rates are altered. Moreover, the drug molecules distribute within the brain ECF with an increasing pattern as time also increases. However, the concentration of drug in Figure 12 is generally higher than the concentration in Figure 11.

When the parameters for specific binding are varied, the amount of drug concentration in specific binding sites (see Figure 19) is smaller than the concentration in nonspecific binding sites (see Figure 20). In addition, when parameters for nonspecific binding are also varied, the concentration of drug in both specific and nonspecific binding sites is almost the same as indicated by Figures 21 and 22, respectively.

## 5. Discussion and Conclusions

In the current study, we have formulated and simulated a mathematical model through which the effect of binding kinetics in the drug distribution within the brain is determined. The model formulated in the current study is an augmentation of the model earlier developed by Vendel et al., 2019 in [2]. In our study, we consider the bidirectional bulk flow of the brain ECF contrary to the model developed by Vendel et al. 2019 in [2] which considers only one direction of the bulk flow of the brain ECF. In addition, we make distinction between specific and nonspecific binding sites along with the subsequent drug distribution in respective binding sites through simulated plots.

The model equations are discretized through the implicit FDM. The discretized equations are then used for simulation from which different plots describing the drug distribution along blood plasma and brain ECF domains are obtained. First, the drug distribution within blood plasma is discussed. Then, different cases of association and dissociation rates in specific and nonspecific binding sites (*k*_*i*on_ and *k*_*i*off_, respectively, for (*i* = 1, 2)) are considered to determine the impacts they impose on drug distribution within the brain ECF.

The findings of this study show how the blood flow rate and BBB permeability influence both drug concentration within blood plasma and the distribution of drug molecules in that domain. The simultaneous increase of the BBB permeability and blood flow rate affect the short term distribution of drug molecules in the blood plasma; yet, with a high BBB permeability, there is an even distribution of drug within the brain. Nevertheless, drug molecules in the brain ECF are influenced by both the permeability of BBB and blood flow rate. However, the concentrations at the binding sites contribute to variations in distribution of drug molecules in the brain ECF.

Contrary to the study by Vendel et al. 2019 [2], the current study investigates the effect of drug binding kinetics in the drug distribution in the brain with variations in binding parameter values. Different cases of varied binding parameter values are considered. The results show that when the higher values for dissociation rates are used while maintaining those for association rates, the gradual decrease in drug concentration within the brain ECF is observed. Also, the drug concentration within the brain ECF becomes much lesser due to drug absorption within the brain ECF. When the alteration of association rates with the unchanged dissociation rates is considered, the concentration peaks of drug within the brain ECF are found to cover different locations within the brain ECF. Moreover, the drug molecules within the brain ECF distribute with an increasing pattern. The results of simultaneous variations in both association and dissociation rates for specific binding sites show that the drug concentration within the brain ECF decreases significantly in relation to an increase in time. Nevertheless, the results of simultaneous variations in both association and dissociation rates for nonspecific binding sites show that the drug distributes in the brain ECF region with the subsequent spatial variations in locations of concentration peaks from the region near *W*_in_ towards the direction of *W*_out_ region.

Furthermore, the current study shows an improved visualization of the impact of binding kinetics together with other parameters associated with both the drug and brain which are involved in the drug distribution process within the brain. However, the model developed in the current study covers a few key components that affect the drug distribution within the brain compared to the components that cover the whole volume of the brain tissue. Hence, this calls for incorporation of other components in 3-dimensional mathematical models of the drug distribution for there to be a more realistic and precise description of drug distribution within the brain.

## Figures and Tables

**Figure 1:** 3D brain unit domain, *W*_in_, *W*_out_ domains, and bulk flow directions.

**Figure 2:** Drug exchange between *W*_pl_ and *W*_ECF._

**Figure 3:** Drug transport in brain capillaries and active transport across the BBB into the brain ECF (a). A cubical lattice (blue) represents a piece of 3-dimensional brain tissue. The cubical lattice is formed of the network of smaller cubic lattices (red). The arrows indicate the bidirectional bulk flow of the brain ECF (b).

**Figure 4:** Drug distribution in blood plasma (*μ*) for *P* = 0.1 × 10^−7^ms^−1^ and *v*_blood_=1 × 10^−6^ms^−1^. The plots (a), (b), and (c) indicate the distribution of drug in the blood plasma (*μ*) for *t* = 2*s*, *t* = 8*s*, and *t* = 14*s*, respectively.

**Figure 5:** Drug distribution in blood plasma (*μ*) for *P* = 0.5 × 10^−7^ms^−1^ and *v*_blood_=1.5 × 10^−6^ms^−1^. The plots (a), (b), and (c) indicate the distribution of drug in the blood plasma (*μ*) for *t* = 2*s*, *t* = 8*s*, and *t* = 14*s*, respectively.

**Figure 6:** Drug distribution in blood plasma (*μ*) for *P* = 2 × 10^−6.9^ms^−1^ and *v*_blood_=1 × 10^−6^*ms*^−1^. The plots (a), (b), and (c) indicate the distribution of drug in the blood plasma (*μ*) for *t* = 2*s*, *t* = 8*s*, and *t* = 14*s*, respectively.

**Figure 7:** Drug distribution in blood plasma (*μ*) for *P* = 0.1 × 10^−7^ms^−1^ and *v*_blood_=1.1 × 10^−5.95^ms^−1^. The plots (a), (b), and (c) indicate the distribution of drug in the blood plasma (*μ*) for *t* = 2*s*, *t* = 8*s*, and *t* = 14*s*, respectively.

**Figure 8:** Drug distribution in brain ECF (*ρ*) for *k*_1on_ = 1 × 10^−1^(*μ*molL^−1^*s*)^−1^, *k*_2on_ = 1 × 10^−2^(*μ*molL^−1^*s*)^−1^, *k*_1off_ = 1 × 10^−2^*s*^−1^, and *k*_2off_ = 1 × 10^−1^*s*^−1^. The plots (a), (b), and (c) indicate the distribution of drug in the brain ECF (*ρ*) for *t* = 2*s*, *t* = 8*s*, and *t* = 14*s*, respectively.

**Figure 9:** Drug distribution in brain ECF (*ρ*) for *k*_1on_ = 1 × 10^−1^(*μ*molL^−1^*s*)^−1^, *k*_2on_ = 1 × 10^−2^(*μ*molL^−1^*s*)^−1^, *k*_1off_ = 5 × 10^−1^*s*^−1^, and *k*_2off_ = 3 × 10^−0.2^*s*^−1^. The plots (a), (b), and (c) indicate the distribution of drug in the brain ECF (*ρ*) for *t* = 2*s*, *t* = 8*s*, and *t* = 14*s*, respectively.

**Figure 10:** Drug distribution in the brain ECF (*ρ*) for *k*_1on_ = 1 × 10^−2^(*μ*molL^−1^*s*)^−1^, *k*_2on_ = 1 × 10^−3^(*μ*molL^−1^*s*)^−1^, *k*_1off_ = 1 × 10^−2^*s*^−1^, and *k*_2off_ = 1 × 10^−1^*s*^−1^. The plots (a), (b), and (c) indicate the distribution of drug in the brain ECF (*ρ*) for *t* = 2*s*, *t* = 8*s*, and *t* = 14*s*, respectively.

**Figure 11:** Drug distribution in the brain ECF (*ρ*) for *k*_1on_ = 0.5(*μ*molL^−1^*s*)^−1^, *k*_2on_ = 1 × 10^−2^(*μ*molL^−1^*s*)^−1^, *k*_1off_ = 2 × 10^−1^*s*^−1^, and *k*_2off_ = 1 × 10^−1^*s*^−1^. The plots (a), (b), and (c) indicate the distribution of drug in the brain ECF (*ρ*) for *t* = 2*s*, *t* = 8*s*, and *t* = 14*s*, respectively.

**Figure 12:** Drug distribution in the brain ECF (*ρ*) for *k*_1on_ = 1 × 10^−1^(*μ*molL^−1^*s*)^−1^, *k*_2on_ = 2.5 × 10^−4^(*μ*molL^−1^*s*)^−1^, *k*_1off_ = 1 × 10^−2^*s*^−1^, and *k*_2off_ = 1.5 × 10^−3^*s*^−1^. The plots (a), (b), and (c) indicate the distribution of drug in the brain ECF (*ρ*) for *t* = 2*s*, *t* = 8*s*, and *t* = 14*s*, respectively.

**Figure 13:** Drug distribution in specific binding sites (*B*_1_) for *k*_1on_ = 1 × 10^−1^(*μ*molL^−1^*s*)^−1^, *k*_2on_ = 1 × 10^−2^(*μ*molL^−1^*s*)^−1^, *k*_1off_ = 1 × 10^−2^*s*^−1^, and *k*_2off_ = 1 × 10^−1^*s*^−1^. The plots (a), (b), and (c) indicate the distribution of drug in specific binding sites (*B*_1_) for *t* = 2 s, *t* = 8 s, and *t* = 14 s, respectively.

**Figure 14:** Drug distribution in non-specific binding sites (*B*_2_) for *k*_1on_ = 1 × 10^−1^(*μ*molL^−1^*s*)^−1^, *k*_2on_ = 1 × 10^−2^(*μ*molL^−1^*s*)^−1^, *k*_1off_ = 1 × 10^−2^*s*^−1^, and *k*_2off_ = 1 × 10^−1^*s*^−1^. The plots (a), (b), and (c) indicate the distribution of drug in non-specific binding sites (*B*_2_) for *t* = 2 s, *t* = 8 s, and *t* = 14 s, respectively.

**Figure 15:** Drug distribution in non-specific binding sites (*B*_2_) for *k*_1on_ = 1 × 10^−1^(*μ*molL^−1^*s*)^−1^, *k*_2on_ = 1 × 10^−2^(*μ*molL^−1^*s*)^−1^, *k*_1off_ = 5 × 10^−1^*s*^−1^, and *k*_2off_ = 3 × 10^−0.2^*s*^−1^. The plots (a), (b), and (c) indicate the distribution of drug in non-specific binding sites (*B*_2_) for *t* = 2 s, *t* = 8 s, and *t* = 14 s, respectively.

**Figure 16:** Drug distribution in specific binding sites (*B*_1_) for *k*_1on_ = 1 × 10^−1^(*μ*molL^−1^*s*)^−1^, *k*_2on_ = 1 × 10^−2^(*μ*molL^−1^*s*)^−1^, *k*_1*off*_ = 5 × 10^−1^*s*^−1^, and *k*_2off_ = 3 × 10^−0.2^*s*^−1^. The plots (a), (b), and (c) indicate the distribution of drug in specific binding sites (*B*_1_) for *t* = 2 s, *t* = 8 s, and *t* = 14 s, respectively.

**Figure 17:** Drug distribution in non-specific binding sites (*B*_2_) for *k*_1on_ = 1 × 10^−2^(*μ*molL^−1^*s*)^−1^, *k*_2on_ = 1 × 10^−3^(*μ*molL^−1^*s*)^−1^, *k*_1off_ = 1 × 10^−2^*s*^−1^, and *k*_2off_ = 1 × 10^−1^*s*^−1^. The plots (a), (b), and (c) indicate the distribution of drug in non-specific binding sites (*B*_2_) for *t* = 2 s, *t* = 8 s, and *t* = 14 s, respectively.

**Figure 18:** Drug distribution in specific binding sites (*B*_1_) for *k*_1on_ = 1 × 10^−2^(*μ*molL^−1^*s*)^−1^, *k*_2on_ = 1 × 10^−3^(*μ*molL^−1^s)^−1^, *k*_1off_ = 1 × 10^−2^s^−1^, and *k*_2off_ = 1 × 10^−1^s^−1^. The plots (a), (b), and (c) indicate the distribution of drug in specific binding sites (*B*_1_) for *t* = 2 s, *t* = 8 s, and *t* = 14 s, respectively.

**Figure 19:** Drug distribution in specific binding sites (*B*_1_) for *k*_1on_ = 0.5(*μ*molL^−1^s)^−1^, *k*_2on_ = 1 × 10^−2^(*μ*molL^−1^s)^−1^, *k*_1off_ = 2 × 10^−1^*s*^−1^, and *k*_2off_ = 1 × 10^−1^s^−1^. The plots (a), (b), and (c) indicate the distribution of drug in specific binding sites (*B*_1_) for *t* = 2 s, *t* = 8 s, and *t* = 14 s, respectively.

**Figure 20:** Drug distribution in non-specific binding sites (*B*_2_) for *k*_1on_ = 0.5(*μ*molL^−1^*s*)^−1^, *k*_2on_ = 1 × 10^−2^(*μ*molL^−1^*s*)^−1^, *k*_1off_ = 2 × 10^−1^*s*^−1^, and *k*_2off_ = 1 × 10^−1^*s*^−1^. The plots (a), (b), and (c) indicate the distribution of drug in non-specific binding sites (*B*_2_) for *t* = 2 s, *t* = 8 s, and *t* = 14 s, respectively.

**Figure 21:** Drug distribution in specific binding sites (*B*_1_) for *k*_1on_ = 1 × 10^−1^(*μ*molL^−1^*s*)^−1^, *k*_2on_ = 2.5 × 10^−4^(*μ*molL^−1^*s*)^−1^, *k*_1off_ = 1 × 10^−2^*s*^−1^, and *k*_2off_ = 1.5 × 10^−3^*s*^−1^. The plots (a), (b), and (c) indicate the distribution of drug in specific binding sites (*B*_1_) for *t* = 2 s, *t* = 8 s, and *t* = 14 s, respectively.

**Figure 22:** Drug distribution in nonspecific binding sites (*B*_2_) for *k*_1on_ = 1 × 10^−1^(*μ*molL^−1^*s*)^−1^, *k*_2on_ = 12.5 × 10^−4^(*μ*molL^−1^*s*)^−1^, *k*_1off_ = 1 × 10^−2^*s*^−1^, and *k*_2off_ = 1.5 × 10^−3^*s*^−1^. The plots (a), (b), and (c) indicate the distribution of drug in specific binding sites (*B*_2_) for *t* = 2 s, *t* = 8 s, and *t* = 14 s, respectively.

**Table 1:** The model parameters, descriptions, values, and units.

Parameter	Description	Value[reference]	Unit
*F*	Drug bioavailability	1 [2]	—
Dose	Concentration of orally delivered drug	0.5 [2]	*μ*mol
*V*_*d*_	Distribution volume	0.2 [2]	*L*
*K*_*a*_	Absorption rate constant	2 × 10^−4^ [2]	*s* ^−1^
*K*_*e*_	Elimination rate constant	5 × 10^−5^ [2]	*s* ^−1^
*r*	Brain capillary radius	2.5 × 10^−6^ [28]	m
*l*_cap_	Inter-capillary distance	5 × 10^−5^ [29]	m
*v*_blood_	Brain capillary blood flow rate	(0.5 − 50) × 10^−6^ [29]	ms^−1^
*T*_*m*−in_	Maximum active influx rate	0.1 × 10^−12^ [assumed]	*μ*mols^−1^
*T*_*m*−out_	Maximum active efflux rate	0.1 × 10^−12^ [assumed]	*μ*mols^−1^
*K*_*m*−in_	Concentration required to attain half of *T*_*m*−in_	1 × 10^2^ [2]	*μ*molL^−1^
*K*_*m*−out_	Concentration required to attain half of *T*_*m*−in_	1 × 10^2^ [2]	*μ*molL^−1^
*D* ^∗^	Effective diffusion coefficient	2.5 × 10^−16^ [20]	m^2^s^−1^
*V*_ECF_	Brain ECF bulk flow velocity	0.5 × 10^−6^ [assumed]	ms^−1^
SA_BBB_	Surface area of the BBB	0.1 × 10^−7^ [assumed]	m^2^
*P*	BBB permeability	10^−10^ − 10^−5^ [2, 8]	ms^−1^
*k*_1on_	Specific association rate constant	10^−4^ − 10^2^ [30]	(*μ*molL^−1^s)^−1^
*k*_2on_	Non-specific association rate constant	10^−6^ − 10^1^ [23]	(*μ*molL^−1^s)^−1^
*k*_1off_	Specific dissociation rate constant	10^−6^ − 10^1^ [30]	s^−1^
*k*_2off_	Non-specific dissociation rate constant	10^−4^ − 10^3^ [23]	s^−1^
*B*_1_^tot^	Total concentration on specific binding sites	5 × 10^−2^ [23]	*μ*molL^−1^
*B*_2_^tot^	Total concentration on non-specific binding sites	5 × 10^1^ [23]	*μ*molL^−1^

## Data Availability

There is no limit on accessing data available in this article. All the data supporting the study are included within the article.
